# Hybrid RGSA and Support Vector Machine Framework for Three-Dimensional Magnetic Resonance Brain Tumor Classification

**DOI:** 10.1155/2015/184350

**Published:** 2015-10-04

**Authors:** R. Rajesh Sharma, P. Marikkannu

**Affiliations:** ^1^Department of IT, Hindusthan College of Engineering and Technology, Coimbatore, Tamil Nadu 641 032, India; ^2^Department of IT, Anna University Regional Centre, Coimbatore, Tamil Nadu 641 046, India

## Abstract

A novel hybrid approach for the identification of brain regions using magnetic resonance images accountable for brain tumor is presented in this paper. Classification of medical images is substantial in both clinical and research areas. Magnetic resonance imaging (MRI) modality outperforms towards diagnosing brain abnormalities like brain tumor, multiple sclerosis, hemorrhage, and many more. The primary objective of this work is to propose a three-dimensional (3D) novel brain tumor classification model using MRI images with both micro- and macroscale textures designed to differentiate the MRI of brain under two classes of lesion, benign and malignant. The design approach was initially preprocessed using 3D Gaussian filter. Based on VOI (volume of interest) of the image, features were extracted using 3D volumetric Square Centroid Lines Gray Level Distribution Method (SCLGM) along with 3D run length and cooccurrence matrix. The optimal features are selected using the proposed refined gravitational search algorithm (RGSA). Support vector machines, over backpropagation network, and *k*-nearest neighbor are used to evaluate the goodness of classifier approach. The preliminary evaluation of the system is performed using 320 real-time brain MRI images. The system is trained and tested by using a leave-one-case-out method. The performance of the classifier is tested using the receiver operating characteristic curve of 0.986 (±002). The experimental results demonstrate the systematic and efficient feature extraction and feature selection algorithm to the performance of state-of-the-art feature classification methods.

## 1. Introduction

Cancers that are most common in children aged 0–14 are brain and central nervous system (CNS) tumors (21%) [1]. A brain tumor is a mass of tissue formed by accumulation of abnormal cells in brain and central nervous system. It is caused by improper metabolic cycle. The cells in human body die over age and are replaced by new cells. But tumor cells grow even though the body does not need them and will not die. The abnormal mass of tissue cells grows uncontrollably intruding normal brain activity. Tumors are categorized as benign (well-defined mass with no cancer cells) and malignant (spreading rapidly to other body parts). Recognition of these tumors from brain, overlapped with dense brain tissues, is very challenging. Any anomalous detection of abnormal tissues results in misdiagnosis of both locus and dimension. Magnetic resonance imaging (MRI) modality is found to best assist tissue contrast for anatomical details and also investigate the mechanisms of the brain by functional imaging towards tumor predictions.

Representation of a 3D data in the form of 2D projected slices results in loss of information and may lead to erroneous interpretation of results [2]. In general, the 2D images cannot precisely convey the complexities of human anatomy and hence interpretation of complex anatomy in 2D images requires special training. Therefore, automatic brain tumor recognition in MRI images is very essential towards diagnostic and therapeutic applications. Hence this paper presents an automatic classification of magnetic resonance images (MRI) of brain under two categories as lesion benign and malignant. Literature studies on texture analysis in biomedical images have directly used the classic methods and hybrid methods [3–6]. In recent years, techniques have been integrated with artificial neural networks (ANNs) and various optimization algorithms to improve the performance.

Ushizima et al. in [6] presented a method employing *k*NN classification to discriminate normal from cognitive impaired patients by describing the white/gray matter (WM/GM) image intensity variation in terms of textural descriptors from gray level cooccurrence matrices (GLCMs). Sharma [7] performed analysis to discriminate glioblastoma multiforme tumor recurrences and radiation injury by first- and second-order texture analysis describing the white/gray matter using a multiparametric characterization of the tissue. Use of 3D texture analysis of T1- and T2-weighted MR images for classification and comparison with the traditional 2D texture analysis approach was employed for classifying pediatric brain tumors [8].

Applicability of 3D texture analysis for extracting additional information from MR images (GCM and run length) and obtaining imperceptible quantitative individual information from MR images of the brain in epilepsy type EPM1 patients was carried out in [9]. Kovalev et al. [10] reported nontrivial classification tasks for pathologic findings in brain datasets. Texture analysis from gradient matrix, run length matrix, autoregressive model, wavelet analysis, and cooccurrence matrices and classification using artificial neural network (ANN) for classifying multiple sclerosis lesion was studied in [11]. Herlidou-Même et al. [12] performed analysis based on 3D histogram, cooccurrence, and gradient and run length matrix parameters for tumor grading.

Li et al. [13] perform classification of gliomas according to their clinical grade employing linear SVMs trained on a maximum of 15 descriptive features. Three-dimensional textural features with an ensemble classification scheme employing a support vector machine classifier to discriminate benign, malignant, and metastatic brain tissues on T1 postcontrast MR imaging were studied in [14]. Gao et al. [15] have performed analysis using 3D local binary pattern (LBP), 3D GLCMs, 3D wavelets, and 3D Gabor textures for brain image retrieval. 3D GLCM and volumetric run length matrix with ELM classifier were proposed for brain tumor tissue classification in [16]. El-Dahshan et al. [17] classified the brain images into normal or abnormal using ANN and *k*-nearest neighbor (*k*NN) classifiers. These include few of the literature studies employed for brain tumor classification and the following section presents the problem statement for the proposed work.

## 2. Brain Tumor Detection Using MRI: Problem Definition

The proposed computer-aided diagnosis system categorizes the tumor detected regions as malignant or benign. It aids the radiologists in recognizing tumor diagnosis. The system in the first phase identifies suspicious lesions at a high sensitivity, which involves a feature extraction process using volumetric analysis on the MRI scans. The second phase aims to detect the tumor and to reduce the number of false positives without decreasing the sensitivity drastically.

The problem of brain tumor detection using MR images consists of the major phases in the proposed classification framework. They are (a) micro-macro feature extraction for each voxel of VOI as 3D volumetric data, (b) optimal feature subset selection using refined gravitational search algorithm from extracted features, (c) the training process enabling SVM classifier for the optimal feature subset selection, and (d) testing of the final framework using leave-one-out validation.  Figure 1 depicts the general flow of the computer-aided design (CAD) classification system.

### 2.1. Materials and Acquisition

320 patient volumes were studied on a 1.5-Tesla MRI machine (Avanto, Siemens Medical Solutions, Germany) with T1w 3D magnetization prepared gradient echo (T1w MPR), obtained from hospitals. The pixel resolution was of 256 × 256 (1 × 1 mm), acquired from the 3D volumes having 128 sagittal slices of 1.25 mm.

### 2.2. Normalization from the ROI

To facilitate reduction of intensity, homogeneity, and removal of artifacts in MR images, a normalization filter, namely, 3D LoG (Laplacian of Gaussian or Mexican Hat) filter, as represented in (1), is employed. The acquired 3D MR volumes are normalized by permitting ripples in both pass band and stop band of the filter. It applies an LoG filter to 3D volumetric analysis. Hence normalization reduces the dynamic range of the intensity values, where feature extraction is made much simpler. As a preprocessing stage, the filter is noted to be a perfect tool for improving the spherical particles enhanced with spots, that is, existence of noisy images in spherical particles. This module is easy to tune, only by selecting the standard deviations in *x*, *y*, and *z* directions [2]. At each voxel with coordinates (*x*, *y*, *z*), the 3D LoG filter is applied to obtain MR image.  Figure 2 represents an MRI case normalized with LoG filter and its histogram analysis is depicted as

(1) LoG=Δgx,y,z=Cx2σx4−1σx2+y2σy4−1σy2+z2σz4−1σz2·e−x2/2σx2−y2/2σy2−z2/2σz2.

### 2.3. Feature Extraction from Statistical Models

Medical images possess a vast amount of texture information relevant to clinical practice. The objective of the feature extraction is to characterize an image to be recognized by measurements, whose values are very similar to those for objects in the same category but very different from those for objects in different categories [18]. The volume of interest (VOI) drawing was performed manually by an expert developing quantifiable radiology in clinical use. Initially the VOI is placed for around 1800 voxels. Further the MR images [19] undergo 3 levels of volume of interest (VOI) selection which are manually placed symmetrically on the left, right, anterior, and posterior hemispheres of both WM and GM.

Feature extraction is the numerical computation of a characteristic or an attribute on a digital image which well describes its texture properties [20]. Any tissue categorization involves quantifiable techniques for detecting various tissues apart from visual interpretation. The objective is to increase the detectability of normal and pathologic tissues. Any tissue categorization can be analyzed by texture analysis. Several methods exist towards texture analysis [21–24].

All possible features are to be extracted towards diagnosing a VOI in the MR image. The extracted feature provides the characteristics of the input type to the classifier by considering the description of the relevant properties of the image into feature vectors. Local features at each point of VOI are to be computed by analyzing the spatial distribution of grey values. Hence a highly defined set of statistical features should be derived to determine the micro-macro texture features. In Figure 3, each of the volumes of interest with an expert level draw is shown. The 3D higher-level extracted features of structure and shape, intensity, variance, and standard deviation should be chosen to preserve the information. The 3D volume measurement is based on the marching cubes volume model of the VOI. The centroid is the 3D *xyz* coordinate of the average Cartesian vectorial position of all voxels within the VOI.

The feature extraction model called Square Centroid Lines Gray Level Distribution Method (SCLGM) for detecting calcifications in 2D mammogram [25] is extended for 3D volumetric analysis of MRI image. The model is augmented with two preexisting feature extraction methods: Run Difference Method (RDM) and the Spatial Gray Level Dependence Method (SGLDM) as in [25] and extended for volumetric analysis of the same.

Along with the 3D gray level cooccurrence matrices (GLCM) [26] and run length matrices [27], the textural features are extracted based on Square Centroid Lines Gray Level Distribution Method (SCLGM) [25] for 3D images. The GLCM computes the textural features using the spatial dependency between the gray level pixel values [26]. The run length matrix quantifies the directional coarseness of a texture for a given VOI. The vectors define the angle and choice of distances. Fine local textures are computed for small values of distances. To ensure global property and coarse textures, distance of *d* ∈ (1, 2,…, *L*/2), where *L* represents the length of VOI, is employed. Hence the five GLCM features and eleven run length features are computed for 13 directions with *d* as defined. In the 3D image mass (VOI) with *n* level gray values, the value of a 3D SCLGM element represents the centroid *C*_*gi*_. It reflects within the centroid the gray levels of voxels *G*(*x*, *y*, *z*) and *G*(*x* + *d*_*x*_, *y* + *d*_*y*_, *z* + *d*_*z*_) and the spatial relationship of displacement vector *d* [28]. This aids in obtaining discriminative features for the VOI in distinguishing between benign or malignant tumor. The detailed featured list is given in the appendix.

In this paper it is intended to extend the Square Centroid Lines Gray Level Distribution Method (SCLGM) feature extraction method for volumetric data, by quantifying the spatial distribution of the square; this approach encodes the spatial interdependency of the cells in all directions. The lowest square includes the segmented area with zero background [25].  Figure 4 depicts the 3D relations between the pixels of each centroid line with directions to provide discriminative information about the mass type. In 2D images, each pixel has 4 directions and 8 neighbors, but when extended to 3D it has 13 directions and 26 neighbors. Similarly, the extension from 4 (centroid lines) for 2D images to 3D is 13 centroid lines (*C*_*i*_) as in Table 1. The centroids are the lines that pass through the square's center point [29]. By obtaining angle *θ*, the object remains perpendicular to the imaging *x*-axis. The center of rotation is based on the object centroid as the center. Using the formula of 3D rotation method, at each centroid, the gray level points are defined as *C*_*gi*_ based on the matrix as given in

(2) xcyczc=cos⁡θ−sin⁡θ0sin⁡θcos⁡θ0001xyzCgi=∀x,y,z:xc=xcos⁡θ−ysin⁡θ;  yc=xsin⁡θ+ycos⁡θ;  zc=z,

where (*x*_*c*_, *y*_*c*_, *z*_*c*_) is the square center, (*x*, *y*, *z*) ∈ VOI, and *θ* ∈ {0,45°, 90°, 135°,…}.

A set of statistics is computed before extracting micro-macro textural features after defining *C*_*gi*_, in SGLDM. The statistics include mean, variance, mean absolute variation, standard deviation, skewness, and kurtosis. 12 features are extracted from each statistical measure. The appendix includes the features extracted. In this work, the 2D texture features as in [25] are extended to 3D volumes of interest, with 12 abovementioned statistics, and 61 three-dimensional texture features are assessed to differentiate textural tissues in MR images from the centroid lines. The features based on centroid as in [25, 30] are calculated for 2D ROI in 4 directions for brain images for comparison. In 3D VOI, all 61 features in 13 directions with an average distance of 1 ⋯ *L*/2 are considered to provide sensitive and specific assessment of tumor.

The textural parameters for the proposed work are calculated in several directions and pixel distances. Mean value for different pixel distances and directions are also computed. Each feature with textural property is used to differentiate the tumor tissues from selected VOI. A set of statistical features are extracted based on 3D Square Centroid Lines Gray Level Distribution Method, 3D GLCM, and 3D run length features. The 61 textural parameters are computed for each centroid as neighbor along 13 directions. All of these texture features are calculated for each VOI.

### 2.4. Optimal Feature Subselection

There arises a need to select most potential features that are highly related to particular classes for classification. This is known as optimal informative feature vector. These features are extracted from an existing feature set to describe the target conceptions of machine learning in classification. The objective is to trace the best minimum subset in the original element set, rather than transforming the data to an entirely new set of dimensions. All extracted features with pooled texture measures are analysed as possibly highly correlated features [16]. Feature subselection model typically incorporates a search strategy for exploring the space of feature subsets [31]. One such model is wrapper based approach which is a procedural searching technique in the defined potential feature subset space. Optimal feature subsets are generated and then evaluated. The specific feature subset is evaluated by training a certain classification model, thus making this approach adaptable to classification algorithm. To reduce the dimension of extracted features, in this research contribution, a heuristic search optimization technique is proposed: refined gravitational search algorithm (RGSA) for continuous optimization.

#### 2.4.1. Classical Gravity Search Algorithm

The classical gravity search algorithm is based on the law of gravity (every particle attracts another particle by means of some gravitational force) and mass interaction [32–34]. In GSA algorithm, the objects (particles) are evaluated with their masses with four features: particle position, inertial mass, active gravitational mass, and passive gravitational mass. Each position of the object provides a solution. The gravitational and inertia masses are navigated with the fitness function of the problem defined. The system in GSA is well defined with *N* mass (agent), where the position of the *i*th agent is denoted as

(3) $$\begin{array}{c} X_{i}=\left(\;x_{i}^{1}\cdots x_{i}^{d}\cdots x_{i}^{n}\;\right)\;\text{for }i=1,2,3,\ldots ,N, \end{array}$$

where *x*_*i*_^*d*^ denotes present position in *d*th dimension of agent *i* and *n* the search space dimension. The force applied between *i*th and *j*th mass at time *t* is given as

(4) $$\begin{array}{c} F_{ij}^{d}=G\left(\;t\;\right)\frac{M_{ai}\left(t\right)\times M_{pj}\left(t\right)}{R_{ij}\left(t\right)+\xi }\left(\;x_{j}^{d}\left(\;t\;\right)-x_{i}^{d}\left(\;t\;\right)\;\right), \end{array}$$

where *M*_*pj*_(*t*) is the active gravitational mass, *M*_*ai*_(*t*) is the passive gravitational mass, *ς* is the small positive constant, *R*_*ij*_(*t*) denotes the Euclidean distance between particle *i* and *j* at time (*t*):

(5) $$\begin{array}{c} R_{ij}\left(\;t\;\right)={\left\|\;x_{i}\left(\;t\;\right),x_{j}\left(\;t\;\right)\;\right\|}_{2}. \end{array}$$

*G*(*t*) represents the gravitational coefficient defined as

(6) $$\begin{array}{c} G\left(\;t\;\right)=G_{0}e^{-\alpha^{t}/T}, \end{array}$$

where *G*_0_ and *α* are constant with *T* being the maximum iteration. The total resultant force exerted on mass *i* in *d* dimension is

(7) $$\begin{array}{c} F_{i}^{d}\left(\;t\;\right)=\overset{N}{\underset{j\in k,j\neq i}{\sum }}r_{j}\cdot F_{ij}^{d}\left(\;t\;\right), \end{array}$$

where *r*_*j*_ is a uniformly distributed random number in the interval [0, 1]. *k* is the set of first *K* agents with the best fitness value to avoid local optimal solutions, where only the *k* best masses, that is, the ones with highest fitness values, will attract the others. Hence by law of motion, the acceleration of the mass *i* at time *t* in *d*th dimension is defined as

(8) $$\begin{array}{c} a_{i}^{d}=\frac{F_{i}^{d}\left(t\right)}{M_{i}\left(t\right)}, \end{array}$$

where *M*_*i*_(*t*) is the inertial mass of particle *i*. The gravitational mass and the inertial mass are updated by the following equations:

(9) MaiMpi=Mii=Mi,i=1,2,…,N,mitfitit−worsttbestt−worstt,Mitmit∑j=1Nmjt,

where fit_*i*_(*t*) denotes the fitness value of mass *i*. For the minimization problem, the worst(*t*) and best(*t*) are given as

(10) bestt=minj∈1,2,…,N⁡fitjt,worstt=maxj∈1,2,…,N⁡fitjt.

In GSA, the updating of velocity and position in each iteration is in accordance with Newton's laws of motion formulized as

(11) vidt+1=randi·vidt+aidt

(12) xidt+1=xidt+vidt+1,

where rand is a random number between the intervals between [0, 1].

#### 2.4.2. Proposed Refined Gravity Search Algorithm (RGSA)

The developed algorithm is based on the interaction of masses steered by the approximation of Newton's laws of gravity and motion. The refined gravity search algorithm is as follows.

**Step 1 .**

Identify the search space.

**Step 2 .**

Generate initial population of *N* agents at random including positions and velocities using uniform distribution.

**Step 3 .**

Fitness evaluation for each agent is calculated in volume of extracted features in 3D axis,

(13) Px,Py,Pz:min⁡:sum_i=1∧i=nxi−Px∧2+yi−Py∧2+zi−Pz∧2,

under the constraint that (*P*_*x*_, *P*_*y*_, *P*_*z*_) lies in the particular VOI of brain region.

**Step 4 .**

Compute* G(t)*,* Best Fitness*, and* Worst Fitness* of the problem.

**Step 5 .**

Calculate the total force in different directions.

**Step 6 .**

Calculate acceleration and velocity.

**Step 7 .**

For each mass *i*, do the following:

Evaluate Fitness_*i*_, Mass_*i*_, Force of Mass_*i*_, Acceleration of Mass_*i*_, and Update Velocity of Mass_*i*_ and find new Position of Agent_*i*_.

**Step 8 .**

Repeat Steps 4 to 7 until a said stopping criterion related to the number of objective function evaluations is reached.

**Step 9 .**

Return the best fitness computed at final iteration as a global fitness and the positions of the corresponding agent at specified dimensions as the global solution of that problem.

To improve the performance of RGSA, Bernoulli updating of *r*_*i*_ in resultant exerted force acting is incorporated on a mass equation (15), where *r*_*i*_ is randomly distributed with

(14) mean=p,variance=p1−p,

where *p* denotes existence of force and 1 − *p* no force. If the force is *f* = 1, there are no movement and no exploration. To further redefine, each mass will be a particle looking towards the new position and velocity updating. Hence Gaussian and logarithmic updating of rand_*i*_ for velocity updating in (11) are defined by

(15) if  randu>0.4then  randi=ln⁡1/randd4else  randi=0.4+0.1×randg,

where rand_*u*_ and rand_*d*_ are uniformly distributed random numbers in the interval [0, 1] and rand_*g*_ is a normally distributed pseudorandom number with mean 0 and standard deviation 1.

Thus, the proposed refined gravity search algorithm provides a well-balanced mechanism in enhancing exploration and exploitation abilities. The performance simulation results show that RGSA attains promising results and outperforms the classical GSA. The rand_*i*_ parameter is used to balance the exploitation/exploration tradeoff. The Gaussian and logarithmic function models are nonstationary functions. Hence the RGSA gives closed-form marginal variances and means. The exploration and exploitation which seek places with high variance and low mean, respectively, are achieved with the use of Bernoulli's function. The acquisition of Gaussian and logarithmic function balances the optimization to determine the next evaluation.  Table 2 represents the parameters employed in refined GSA for brain tumor classification.

### 2.5. SVM Classification for Tumor Recognition

Classification is a procedure for sorting pixels and assigning them to specific categories. It is about predicting unknown class of an observation. Statistical analysis involves relationship with the variables to a model developed. Models include neural networks, *k*-nearest neighbor, AdaBoost, tree classifiers, and many more. Techniques for modeling data and analysis can be categorized as supervised and unsupervised learning. Amongst all, the support vector machines outperform various state-of-the-art classifiers in medical image classification as an efficient training algorithm for large scale problems. SVM has been comprehensively used as a classification tool in domains of image analysis and real-world problems.

In classification, if the characteristics or attributes (predictor variable) of a class are known, individual objects might be identified as belonging or not belonging to that class. This transformed attribute used to define the hyperplane is called a feature. Feature selection stage chooses the most optimal attributes. A set of features that labels one instance (i.e., a row of predictor values) is called a vector. SVM technique separates the identified classes with a particular hyperplane to the nearest point in the dataset [35, 36]; that is, the cluster of vectors of positive examples of one case of the target lies on one-half of the plane, with the other case on the other side as negative examples as denoted in Figure 5. The vectors near the optimal hyperplane with maximal distance of the nearest samples from each class are termed as support vectors [37].

The basic principle of SVM is to search for optimal hyperplane with maximal distance of the nearest samples from each class. Consider the images to be classified as *N*, where *n* = 1, 2,…, *N*, and their respective weighted features are [*f* ^∧^1, *f* ^∧^2,…, *f* ^∧^ *N*]. The aim is to classify these images into two classes, that is, lesion benign and malignant, binary classification with the help of kernel function [37, 38]. Consider the training data of the form *D* = {(*x*_1_, *y*_1_),…, (*x*_*m*_, *y*_*m*_)}, where *m* is the number of training samples, and associated output *y*_*i*_ ∈ {+1, −1} as class label and the linear classification function as

(16) $$\begin{array}{c} f\left(\;x\;\right)=v,x+b \end{array}$$

with *v* being a weighted vector and *b* a scalar bias value.

The optimal classifying plane and the support vectors are depicted in Figure 5. The describing optimal separating hyperplane is given by

(17) $$\begin{array}{c} \langle \;v,x\;\rangle +b=0. \end{array}$$

The space between the optimal plane encirclement is equal to 2/‖*v*‖, where ‖*v*‖ is the Euclidean norm of *v*. In order to maximize the margin,

(18) Minimize: 12·v·v′+Csubject to: viv′·zi+b≥1−ξi, ∀i,

where *ξ*(≥0) is the slack variable and *C* is the regularization parameter. The Lagrange function is defined as

(19) $$\begin{array}{c} L=\frac{1}{2}{\left\|\;v\;\right\|}^{2}-\overset{m}{\underset{i=1}{\sum }}\alpha_{i}y_{i}\langle \;v,x\;\rangle +b+\overset{m}{\underset{i=1}{\sum }}\alpha_{i}, \end{array}$$

where the original space is projected into a high dimension space to construct an optimal hyperplane with the dual optimization problem obtained to maximize

(20) vα=∑i=1mαi−12∑i=1 m∑ j=1mαiαjyiyjKxi,xsubject to:  ∑i=1myiαi=0,0≤αi≤C,  ∀i,

with *α*_1_ ⋯ *α*_*m*_ being the nonnegative Lagrangian multiplier. The classification function is defined as

(21) $$\begin{array}{c} y=\mathrm{sign}\left(\;v\cdot z+b\;\right)=\mathrm{sign}\left(\;\overset{m}{\underset{i=1}{\sum }}\alpha_{i}\cdot y_{i}K\left(\;x_{i},x\;\right)+b\;\right). \end{array}$$

Here the radial basis function *K*(*x*, *z*) = exp⁡{−‖*x* − *z*‖^2^/2*σ* ^2^} is used to construct the SVM classifier. When the functions *f*(*x*) > 0, the input vector *x* belongs to one class (benign); if *f*(*x*) < 0, input vector *x* belongs to the other (the malignant) [39]. The SVM parameters [40] *C* and *σ* are to be optimized during classification. The fitness function of the network is given by

(22) $$\begin{array}{c} \text{fitness}=\theta \times SVM\;\;\text{accuracy}+\left(\;1-\theta \;\right)\times {\text{featuresel}}^{-1}, \end{array}$$

where SVM  accuracy is classification accuracy of SVM; featuresel is the number of selected features; and *θ* is the weight of SVM accuracy, which is used to adjust the proportion of SVM  accuracy and featuresel; it is set as 0.7. Equation (22) ensures high fitness if SVM  accuracy is high and featuresel is low.  Table 3 shows the various parameters assigned for implementing SVM classifier for proposed application.

In this paper, along with the proposed RGSA, the SVM classifier is used for brain tumor detection. The realized SVM classifier avoids overtraining and performs better generalization. The classifier is evaluated for performance and the results are compared with a standard BPN and *k*NN classifier.

## 3. Experimental Results and Discussion

For implementing the proposed methodologies, the test data considered is of 320 real-time brain volume images. Leave-one-out classification (LOO) method is used to build the classifier with training and testing datasets. LOO approach is a special case of the *k*-fold cross-validation where *k* represents the size of the data; hence in each step, a single case or sample is used to assess the error rate. After normalization the volumetric features were extracted significantly towards correct diagnosis of cancerous and noncancerous tissues. The variations of microstructural features are obtained by statistical features analysis on 3D VOI images. Out of 14 GLCM features, six common volumetric features had equal discriminatory power of the gray level cooccurrence matrices computed for 3D VOI of images [26]. The features are selected to differentiate the image tissues to discern malignant and benign cancer. Further, the eleven run length volumetric (statistical) features were generated for number of gray levels *G* and maximum run length with thirteen directions [27].

The extended volumetric Square Centroid Lines Gray Level Distribution Method for volumetric images enhanced the classification accuracy of the diagnosis system. Based on the thirteen centroid lines, 61 features are extracted; each was represented by thirteen vectors, that is, *C*_*θ*_ vectors comprising the nonzero gray level value.

The proposed methodology extracted a total of 77 features. In this case, refined gravitational search algorithm (RGSA) is applied for feature selection; the obtained selected features are ranked with respect to the number of occurrences and fitness function criteria. 28 features are observed to be the most prominent ranked optimal subselected features out of which 16 features comprised from the 3D extended gray level squared centroid method are extracted [25]. The histogram of the entropy feature is depicted in Figure 6. The blue curves in Figure 6 represent benign distribution and malignant distribution in the volume of interest. Out of the 28 features subselected which aid the discrimination capability towards benign and malignant tumor detection, the histogram of one such attribute (entropy) for the two classes is depicted in Figure 6.  Figure 7 represents the features extracted in the model.  Figure 8 shows tumor segmentation of real-time dataset along with expert segmentation. The comparison of 2D GLCM, 3D GLCM+RLM, and proposed centroid model is presented. The proposed model outstands with respect to other models.

On analysis of global classifier, the classification is performed and compared with BPN, *k*NN, and SVM classification algorithms. The SVM method was best suited with overall classification accuracy of 98.3%, sensitivity of 92.9%, and specificity of 94.3%. The textural features were computed for 2D region of interest (ROI) for the same dataset. Out of seventy-seven features, thirty-nine features were selected to be optimal, reporting the classification accuracy to be 91.5%. Hence 3D VOI analysis showed a better discrimination towards cancer analysis (benign and malignant) cross-validated by leave-one-out validation.

The evaluation of the classifier depends on the misclassification rate. The sensitivity and specificity values are used to compute misclassification rate and success of the diagnostic system of the classifier. Sensitivity is the probability of positive diagnosis test with true cases of tumor defined as

(23) $$\begin{array}{c} \text{Sensitivity}=\frac{\text{TP}}{\text{TP}+\text{FN}}. \end{array}$$

Specificity is defined as the probability of a negative diagnosis test with false case of tumor defined as

(24) $$\begin{array}{c} \text{Specificity}=\frac{\text{TN}}{\text{TN}+\text{FP}}, \end{array}$$

where TP is the number of true positives: number of tumor cases correctly classified; TN is the number of true negatives: number of healthy cases correctly classified; FP is the number of false positives: number of healthy cases classified as tumors; and FN is the number of false negatives: number of tumor cases classified as healthy [41]. RMSE (root mean square error) is the difference between predictions and corresponding observed values are each squared and then averaged over the sample [37]. Mean absolute error (MAE) is a linear score which computes the average magnitude of the errors in a set of predictions with all individuals giving equal weight age. The MAE is the average over the verification sample of the absolute values of the differences between predictions and the corresponding observation. The observed values of RMSE and the MAE parameters, in case of SVM for both training and testing, are proven as the optimal with lowest values.  Figure 9 depicts the simulation results of various classifiers.  Table 4 shows the performance of the classifiers.

The accuracy of the model depends on discrimination between true negatives and false negatives. Accuracy is measured by the area under the ROC curve. The area under a ROC curve (*A*_*z*_ value) obtained by the proposed methodology is 0.986 based on a leave-one-out test in identification of 320 datasets. The best classifier is the support vector machine, since its ROC curve is located at the top of Figure 10. The AUC, as a general summary measure of the classifiers performance, is AUC = 0.96 for the support vector machine, AUC = 0.90 for the *k*NN, and AUC = 0.83 for the backpropagation network (BPN).

The optimal operating points of the three classifiers are computed at (FP = 0.15, TP = 0.94) for the SVM, (FP = 0.20, TP = 0.89) for the *k*NN, and (FP = 0.42, TP = 0.84) for the BPN, where the numbers inside the brackets indicate the false positive (FP) and the true positive (TP). These three points are the maximum optimal (FP, NP) points when the three classifiers are trained with the full training dataset. To investigate the significance of the three classifiers, a Wilcoxon signed-rank test, a nonparametric test, is applied to determine the significance between the texture measure combinations. In case of SVM, the test shows a statistical significant difference on a significance level of 0.05 (i.e., *p* < 0.05), whereas, for BPN and *k*NN, in both cases the difference in AUC of the ROC is statistically significant with *p* = 0.793.  Table 5 shows the average results computed for the proposed SVM classifier with that of BPN and *k*NN with respect to specificity, sensitivity, accuracy, ROC, and mean square error. It is well proved in Table 5 that the developed SVM classifier achieves very minimal mean square error of 0.015 in comparison with that of the earlier classifier models. It also possesses highest level of accuracy, proving its efficiency.

The support vector machine classifier, which classifies the patients to the class which is most probable, will result in one patient data being wrongly classified, leading to a correct classification rate of 98% for the 30 patients sample dataset. This is visualized in Figure 11, where a scatter plot of the classification for the 30 patients is shown. Similarly Figures 12 and 13 indicate the scatter plot of both *k*NN and BPN classifiers, respectively. The circles indicate a patient with malignant tumor prognosis, while the pluses are patients with benign cancer prognosis. The line marks the 50% error or correct classification rate. The axis in the scatter plot diagram is the number of images, for each patient that is classified into the two classes, with benign prognosis on the *y*-axis and malignant tumor prognosis on the *x*-axis.

The proposed refined gravitational search algorithm creates a set of solutions over single result to overcome the trap of local optimum. The exploration feature enhances the RGSA algorithm as a promising method for feature selection over a high dimension space.  Table 6 shows the performance analysis of the classifiers using the already existing two-dimensional approaches and the proposed algorithm. From Table 6 it is noted that the proposed 3D approach with the SVM classifier achieves better accuracy in comparison with that of BPN and *k*NN classifiers.  Figure 14 indicates the average rate of both algorithms, traditional GSA and proposed RGSA. Improved result on search space is found to be in RGSA method using Bernoulli's updating in Figure 15.

In this research paper, the proposed RGSA is applied to select features and optimize SVM parameters simultaneously. GSA is a powerful global optimization algorithm but leads to exploration and exploitation tradeoff as other optimization algorithms [40]. Therefore, the velocity updating of RGSA improves the search space dimension. The experimental result shows that RGSA is of superior performance in feature selection optimization and SVM classification. Hence the proposed RGSA-SVM improves the classification accuracy by minimal optimization of the feature sets and SVM parameters simultaneously.

## 4. Conclusion

This paper presented a new approach towards identification of the brain regions responsible for brain tumor employing an improved version of gravitational search optimization algorithm for optimal feature selection and high dimensional SVM classifier. The feature extraction stage is an extension of the 3D VOI volumetric model using squared gray level centroid method combining the cooccurrence and run length features which resulted in promising outputs. Thus, it is inferred that the best performance of SVM classifier resulted in better testing performance with a lower error and higher accuracy.

The present work will aid in analyzing pathologies and increasing the physician towards reliable diagnosis. The proposed texture analysis model provides an automated tumor discrimination process through the optimum features which best characterizes MRI brain benign and malignant tumors. The proposed methodology could be extended to classify different grades of cancer (e.g., glioma and meningioma) and degree of malignancy.

## Figures and Tables

**Figure 1:** Framework of the proposed CAD classification model.

**Figure 2:** Normalized 3D LoG filter operation.

**Figure 3:** Expert level draw on each volume of interest (VOI).

**Figure 4:** Three-dimensional directions drawn towards a VOI.

**Figure 5:** SVM classification.

**Figure 6:** Histogram analysis of entropy feature set.

**Figure 7:** Features extracted from the integrated 3D approach.

**Figure 8:** Tumor segmentation results on real-time datasets: (a) original MRI segmentation by (b) expert, (c) 2D GLCM+2D RLM+2D centroid model, and (d) proposed 3D GLCM+3D RLM+3D centroid model.

**Figure 9:** Classification accuracy for the considered classifiers.

**Figure 10:** ROC curve for various classifiers.

**Figure 11:** Scatter plot of real-time sample set (30) on SVM classifier for benign and malignant tumor in real-time image dataset. Here “∘” denotes tumor malignant prognosis and “+” denotes patients with benign tumor prognosis.

**Figure 12:** Scatter plot of real-time sample set (30) on *k*NN classifier for benign and malignant tumor in real-time image dataset. Here “∘” denotes tumor malignant prognosis and “+” denotes patients with benign tumor prognosis.

**Figure 13:** Scatter plot of real-time sample set (30) on BPN classifier for benign and malignant tumor in real-time image dataset. Here “∘” denotes tumor malignant prognosis and “+” denotes patients with benign tumor prognosis.

**Figure 14:** Feature selection improvement of proposed RGSA and GSA.

**Figure 15:** Feature selection improvement of proposed RGSA and traditional GSA.

**Table 1:** Thirteen directions and offset for 3D images.

Sl. number	Offset	Degree, direction (θ, ϕ)
1	0, 1, 0	0°, 0°
2	−1, 1, 0	45°, 0°
3	−1, 0, 0	90°, 0°
4	−1, −1, 0	135°, 0°
5	0, 1, −1	0°, 45°
6	0, 0, −1	0°, 90°
7	0, −1, −1	0°, 135°
8	−1, 0, −1	90°, 45°
9	1, 0, −1	90°, 135°
10	−1, 1, −1	45°, 45°
11	1, −1, −1	45°, 135°
12	−1, −1, −1	135°, 45°
13	1, 1, −1	135°, 135°

**Table 2:** Parameters of refined GSA (RGSA).

RGSA parameters	Parametric values
Number of agents	100
Maximum number of iterations (stop criteria)	500
Objective function	Minimization
*G*_*o*_	100

**Table 3:** Parameters of SVM classifier.

SVM parameters	Parametric values
Simulation time	50 ms
Bias value	1
Weights assigned	Random initialization
Number of selected features	0.7

**Table 4:** Performance of the classifiers.

Classifier	Training stage efficiency				Validation stage efficiency			
	Mean	STD	RMSE	MAE	Mean	STD	RMSE	MAE
Proposed SVM classifier	100	0	0.004	0.231	98.45	4.4	0.101	0.281
*k*NN [17]	97.34	0.75	0.125	102.33	90.12	5.6	0.183	138.33
BPN [17]	98.34	1.01	0.128	155.45	89	5.9	0.175	177.32

**Table 5:** Average results on the 3D feature extraction model for various classifiers on real-time 320 patient data volumes.

Classifier	Specificity %	Sensitivity %	Accuracy %	ROC (*A*_*z*_)	Mean square error
BPN [17]	68.17	89.58	88.85	0.89	0.21
*k*NN [17]	76.19	91.84	91.14	0.93	0.10
Developed SVM classifier	**95.0**	**98.94**	**98.4**	**0.99**	**0.015**

**Table 6:** Performance analysis of classifiers and feature extraction, both 2D and 3D.

Texture analysis	Classifier	Accuracy % w/o feature selection	Accuracy % with feature selection
	BPN	72.45	81.2
2D GLCM + 2D RUN LENGTH + 2D SGLDM [25]	*k*NN	84.34	89.45
	SVM	89.55	91.02

Proposed 3D GLCM + 3D RUN LENGTH + 3D SGLDM	BPN	81.65	88.85
	*k*NN	89.55	91.14
	SVM	90.78	98.4

**Table 7:** 

Features	Formula
Run length features	
Short Run Emphasis (SRE)	$\frac{1}{n_{r}}\sum_{i=1}^{M}\sum_{j=1}^{N}\frac{p\left(i,j\right)}{j^{2}}$
Long Run Emphasis (LRE)	$\frac{1}{n_{r}}\sum_{i=1}^{M}\sum_{j=1}^{N}p\left(i,j\right)*j^{2}$
Low Gray Level Run Emphasis (LGRE)	$\frac{1}{n_{r}}\sum_{i=1}^{M}\sum_{j=1}^{N}\frac{p\left(i,j\right)}{i^{2}}$
High Gray Level Run Emphasis (HGRE)	$\frac{1}{n_{r}}\sum_{i=1}^{M}\sum_{j=1}^{N}p\left(i,j\right)*i^{2}$
Short Run Low Gray Level Run Emphasis (SRLGE)	$\frac{1}{n_{r}}\sum_{i=1}^{M}\sum_{j=1}^{N}\frac{p\left(i,j\right)}{i^{2}*j^{2}}$
Short Run High Gray Level Run Emphasis (SRHGE)	$\frac{1}{n_{r}}\sum_{i=1}^{M}\sum_{j=1}^{N}\frac{p\left(i,j\right)*i^{2}}{j^{2}}$
Long Run Low Gray Level Run Emphasis (LRLGE)	$\frac{1}{n_{r}}\sum_{i=1}^{M}\sum_{j=1}^{N}\frac{p\left(i,j\right)*j^{2}}{i^{2}}$
Long Run High Gray Level Run Emphasis (LRHGE)	$\frac{1}{n_{r}}\sum_{i=1}^{M}\sum_{j=1}^{N}p\left(i,j\right)*i^{2}*j^{2}$
Gray Level Nonuniformity (GLNU)	${\frac{1}{n_{r}}\sum_{i=1}^{M}\left(\sum_{j=1}^{N}p\left(i,j\right)\right)}^{2}$
Run-Level Nonuniformity (RLNU)	${\frac{1}{n_{r}}\sum_{j=1}^{N}\left(\sum_{i=1}^{M}p\left(i,j\right)\right)}^{2}$
Run Percentage (RPC)	$\text{RPC}=\frac{n_{r}}{p\left(i,j\right)*j}$

GLCM features	
Entropy	∑_*i*_^*M*^∑_*j*_^*N*^ *P*[*i*, *j*]log⁡*P*[*i*, *j*]
Homogeneity	$\sum_{i=1}^{M}\sum_{j=1}^{N}\frac{p\left[i,j\right]}{1+|i-j|}$
Contrast	∑_*i*_^*M*^∑_*j*_^*N*^(*i* − *j*)^2^ *P*[*i*, *j*]
Energy	∑_*i*_^*M*^∑_*j*_^*N*^ *P* ^2^[*i*, *j*]
Correlation coefficient	$\sum_{i=1}^{M}\sum_{j=1}^{N}\frac{\left(i-\mu \right)\left(j-\mu \right)P\left[i,j\right]}{\sigma^{2}}$

## Appendix

### List of Volumetric 3D Features Extracted

See Table 7.
